The article "Application of Multiple Regression Analysis Model in Table Tennis Competition" was retracted in 2023. Reasons: unreliable results or conclusions; concerns about the data; concerns about the peer review; concerns about the citations.

# Application of Multiple Regression Analysis Model in Table Tennis Competition

**DOI:** 10.1155/2022/6748465

**Published:** 2022-08-01

**Authors:** Yuanjing Li, Yi Wang, Nan Gu, Yecheng Cao, Minghui Ye

**Affiliations:** ^1^The Department of Physical Education, Hebei University of Economics and Business, Shijiazhuang 050061, China; ^2^Competitive Sports Institute of Beijing Sport University, Beijing 100084, China; ^3^Department of Physical Education, Shijiazhuang University, Shijiazhuang 050035, China; ^4^Sports Training Department of Hebei Institute of Physical Education, Shijiazhuang 400067, China

## Abstract

Since the table tennis mixed doubles competition was officially listed as the Olympic Games, the players around the world paid more attention to the project. In this background, the 20 mixed doubles finals were used in the literature, video observation, and analysis of multiple regression. From the receiving point of view, the score difference between men and women is not very great, but female players may be more consistent. The contribution of male and female scores to the game is more effective than model 1 and model 2 for different rounds. Therefore, model 2 is more efficient in the analysis of high-level table tennis competitions. Multiple regression model can be used to analyze and predict table tennis singles, doubles, and mixed doubles games, which we will see more and more in future research results.

## 1. Introduction

Multiple regression analysis refers to the statistical analysis method in which one variable is regarded as dependent variable and other one or more variables as independent variables, establishing linear or nonlinear mathematical model quantity relationship between multiple variables and using sample data for analysis. In addition, there are multiple regression analysis discussing the linear dependence of multiple independent variables and multiple dependent variables, called multiple multiple regression analysis model (or many-to-multiple regression). The relationship between variables is often studied when processing measured data. The relationships between the variables are generally divided into two categories. One is to fully determine the relationship, that is, the functional relationship; one is the correlation, that there is a close connection between variables, but cannot find the value of the other variable (question 1). The task of regression analysis is to use mathematical expressions to describe the relationship between the relevant variables. The basic idea of regression analysis is that although there is no strict, deterministic functional relationship between the independent variables and the dependent variables, we can try to find the mathematical expression forms that best represent their relationship. The study of the regression of a dependent variable and two or more independent variables, also known as multiple linear regression, is the law reflecting that the number of a phenomenon or things changes accordingly according to the change of multiple phenomena or the number of things. Multivariate regression is a statistical method to establish linear or nonlinear mathematical model relations among multiple variables. The application of multiple regression models in sports is not uncommon [1–5]. However, the application of multiple regression analysis in table tennis competition, especially in the practice of table tennis technology and tactics, is not very much.

In order to implement article 11 of the Olympic 2020 agenda, in June 2017, the IOC officially established the table tennis mixed doubles event (mixed doubles event) as the event of the 2020 Tokyo Olympic Games. This is another major move by the IOC after changing doubles in table tennis to teams at the 2008 Beijing Olympics. The main purpose of the reform is to allow men and women to increase the competition and further increase the influence of table tennis around the world. The International Table Tennis Federation stipulates that each association at the Tokyo Olympics can only send a pair of mixed doubles players, which gives many foreign athletes hope of winning medals or even gold medals, thus prompting them to prepare more actively for mixed doubles.

By reviewing the literature, this paper found that only a few scholars have studied table tennis doubles and mixed doubles, most of which are the technical and tactical analysis of pairs of mixed doubles players. Although the evaluation methods of table tennis skills and tactics are increasing in the world [6–14], they are all based on the three-stage index evaluation method proposed by the Chinese scholar Wu Huanqun. In addition, there are some documents on the construction of other network projects, such as technical and tactical analysis models such as tennis [15–19]. However, in the technical and tactical evaluation of mixed doubles players, the method is to treat a pair of players as a whole. In the mixed doubles competition, the speed, rotation, landing point, strength, and rhythm between men and women players are quite different, and the technical and tactical characteristics of the rotation of doubles are also different. Therefore, this paper applies the research method of multiple regression analysis to deeply investigate the unique technical and tactical rules of mixed doubles competition, which can provide a new research perspective and theoretical reference for the development of mixed doubles competition in China. Coaches and athletes from all over the world can fit in and analyze their mixed doubles according to the research methods of this study, which can better evaluate the technical and tactical performance of mixed doubles athletes in the competition, enrich the technical and tactical theory of table tennis, and promote the status of mixed doubles in table tennis.

## 2. Methods and Data

### 2.1. Study Subjects

According to the needs of this research, through web of science and other websites with table tennis and multiple regression as keywords, we obtained more than 20 related articles of table tennis competition to analyze and understand the current development status of table tennis technology and tactics research in China.

This study consisted in the mixed doubles competition. Table tennis mixed doubles is a combination of men and women, each 1 athlete, the players in order of the ball, each four players according to the rules, in 8 points, each has 1 round, 1 round, this hair round set is according to the gender of the winner, respectively, called “male, male, male, male, female, female, female, female” eight rounds, as shown in the figure, record the gain and loss of each round. Eight rounds of mixed doubles competition are shown in Figure 1.

### 2.2. Video Recording Observation Method

This study observed and analyzed the world high-level table tennis mixed doubles competition in the past 5 years. The specific competition information is shown in Table 1.

### 2.3. Mathematical Modeling Method

Mathematical modeling is to build a mathematical model according to the actual problems, to solve the mathematical model, and then to solve the actual problems according to the results. When it is necessary to analyze and study a practical problem from a quantitative perspective, people should establish mathematical models with mathematical symbols and language on the basis of in-depth investigation and research, understanding object information, simplifying assumptions, and analyzing internal laws. Nearly more than half a century, with the rapid development of computer technology, the application of mathematics not only in engineering technology, natural science, and other fields plays a more and more important role, and with unprecedented breadth and depth to the economy, management, finance, biology, medicine, environment, geology, population, transportation, and other new fields, the so-called mathematical technology has become an important part of contemporary high and new technology.

## 3. Statistics of the Data of 2 Receiving Rounds

It was observed that the mixed doubles competition is divided into two types of serving and receiving serve, and serve is divided into two categories: male and female athletes serving, and receiving serve is divided into two categories: male and female athletes receiving serve. The score rate and average score rate were analyzed below. The specific formula is as follows:

(1) $$\begin{array}{c} \text{Male}\left(\text{female}\right)\text{serve score rate}=\frac{\text{male}\left(\text{female}\right)\text{serve round total score}}{\text{the team's service round total score}},\\ \text{Male}\left(\text{female}\right)\text{reception score rate}=\frac{\text{male}\left(\text{female}\right)\text{reception round total score}}{\text{the team serve round total score}},\\ \text{Average score rate}=\frac{\left(\text{score rate per game}\right)}{\text{total number}}. \end{array}$$

### 3.1. Data Statistics of Service Rounds

The scores of the male and female players in the service round are shown in Table 2. We can see the following from the table: in the rounds of male athletes serving, the average score rate is 44.7%, and the average score loss rate is 48.46%. In the rounds of female athletes, the average score rate was 55.30, and the average score loss rate was 51.54%. It can be seen that the average scoring rate and loss rate in the rounds of male serve are small and larger in the rounds of female serve. So, it is more difficult to directly indicate which of both men and women contribute more.

The scores of the male and female players in the receiving round are shown in Tables 2 and 3. We can conclude that in the rounds of male athletes, the average score rate is 52.73%, and the average score loss rate is 47.05. In the receiving rounds of female athletes, the average score rate was 47.27%, and the average score loss rate was 52.95%. It can be seen that the average scoring rate and loss rate are larger in the rounds and larger. To some extent, it can show that the male athletes contribute more than the female athletes. The contribution rate of female athletes was 40.57% of male athletes and 59.43% of female athletes, and female athletes were greater than male athletes.

For the rounds of the winners and losers, as shown in Figure 2, the data illustrate the comparison of the gains and losses in each round.

### 3.2. Comparison of the Gains and Losses of Male and Female Athletes in the 8 Rounds

There are eight rounds in mixed doubles: male-s-male, male-s-female, female-s-male, female-s-female, male-r-male, male-r-female,Women-r-men, and women-r-women. The contribution of male and female athletes to performance over eight rounds is similar to the analysis above. The scoring and loss rates of male and female athletes are shown in Figure 3. It can be seen that the contribution rate of male athletes is 62.03% and that of female athletes is 37.97%, with male athletes greater than female athletes. The contribution rate of female athletes was 58.95%, and that of female athletes was 41.05%, and male athletes were greater than female athletes. The contribution rate of male athletes was 61.90% and that of female athletes was 38.10%, and male athletes were greater than female athletes, as shown in Figure 3.

#### 3.2.1. Loss and Loss of Service Round

In the rounds of “male hair,” the board order is board 1-male, board 3-female, board 5-male, male athletes scored 147 in 20 innings, and female athletes scored 90, less than the “male hair” round, board 1-female, board 3-male, board 5-female, male athletes scored 168 and female athletes scored 117, less than male athletes.

The scoring rate of women in the female rounds is 61%, which belongs to the obvious relative advantage round. The hitting order is the women's serve, the men's third cricket order, the women's fifth cricket order, the women's reception order, the men's fourth cricket order, and so on. As shown in Figure 3, the score rate of women's serve accounted for 17% of the round score, the men's score rate on the 3rd board was 53%, the women's 5th board was 18.9%, the score rate of men after the 5 boards was 7.4%, and the score rate of women after the 5 boards was 4%. Figure 3 visually shows that the scores of this round are mainly focused on the top 3 boards, especially the men's third board.

The scoring rate of women's rounds is 56.9%, which is also the stronger round. The hitting order is the same as that of women's rounds. The difference is that the opponent's hitting order becomes men's reception and women's fourth cricket strike. The round was as follows: women's serve scored 23.3%, men's 34.6%, and women's 51.8%. It can be found by the board order scoring rate that although the scoring rate of men in this round has decreased slightly, it is still the main scoring time. The scoring timing of women's serve and men's connecting rounds are relatively similar, and the tactics are related. Grasping the women's serve round has an important role in winning the game.

Serve attack tactic is a main scoring method of table tennis competition. After the women's serve, the men create a great deterrent to the other side's serve, thus increasing the pressure on the opponent to receive the serve. In addition, the man's third board attack and control ability is strong, once can attack first, the formation of an active situation to the opponent's oppression, not only can directly score, but also for the woman's fifth board connection and even the initiative after the 5th plate to lay a foundation. The main scoring points of women's serve rounds come from the hair and rush period, which shows that the quality and stability of women's serve and men's connection should be continuously strengthened in the mixed doubles training, and full use of the advantages of women's serve rounds should be made in the competition to occupy the initiative of the competition.

The scoring rate of men's round is 57.7%, which belongs to the relatively dominant round. In the order of male and female rotation, the board order is men's serve, women's serve, women's third cricket, men's fifth cricket, the opponent hitting order is men's receiving serve, women's fourth cricket, and so on. The effect of the round was as follows: men's serve was 22.4%, women's 33.6%, men's 32.3%, men's 9.6%, and women's 4.1%. Through the scoring rate, it can be found that the scoring timing of this round changed compared with the women's serve round. The scoring rate of women's third board in the round decreased by 14% and 19.8% compared with that of men's third board, respectively, while the scoring rate of men's fifth board was 13.6% and 16.5% of women's fifth plate in the other two rounds. The above data show that the fifth board is an important scoring time for this round, so the important tactical form of “3 and 5 board connection” should be fully utilized and grasped in the tactical training and competition of this link.

The scoring rate of men's and women's rounds was 52.8%, the lowest scoring rate in mixed doubles. The hitting order was the same as that of men's rounds, and the opponent changed to women's receiving and men's fourth cricket. The plate order scores in this round are as follows: men's serve scored 31.3%, women's third board 44.4%, men's fifth board 19.6%, men's five board 6%, and women after the five board 5%. In this round, the highest scoring rate is the four serve rounds. Objectively speaking, the quality of men's serve is a relatively great threat to women. The scoring rate of the third board of this round was 9.6% higher than that of men's round, once again indicating the threat of men's serve to women's return. However, the scoring percentage of the fifth plate in this round was relatively small, indicating that the return quality of the opponent's fourth plate limited the men's direct score to some extent. The scoring pattern presented in this round is very consistent with the competitive characteristics of the mixed doubles competition. The uncertainty caused by the rotation of shots between male and female players changes with each cricket shot, and the situation in the competition process changes rapidly. Mixed doubles events should constantly strengthen the individual ability, especially women's active attack and men's defense ability, so as to better form a continuous attack, combination attack, antiattack transformation, and offensive and defensive conversion.

#### 3.2.2. Loss and Loss of Receiving and Serving Round

The contribution rate of gain and loss of receiving rounds is shown in Figure 4.

Figure 4 shows the contribution of receiving round, “male” rounds, board order for plate 2-male, 4-female, 6-male, male athletes in 20 total score 142, female athletes scored 89, less than male; and “male” round, board order is the second board-female, fourth-male, sixth board-female, male athletes in 20 scored 87, female athletes score 127, more than the male athletes.

The contribution of receiving round, “male” rounds, board order for plate 2-male, 4-female, 6-male, male athletes in 20 total score 142, female athletes scored 89, less than male; and “male” round, board order is the second board-female, fourth-male, sixth board-female, male athletes in 20 scored 87, female athletes scored 127, more than the male athletes.

The scoring rate of female receiving rounds was 52.8%, and the scoring rate was higher than that of male and female receiving rounds. It was different from the two most relative advantage rounds, so it was not defined as relative advantage rounds or relatively weak rounds. The round is women's 2, men's 4, women's 6, men's serve, women's 3, men's 5, and so on. The gains and losses of the first 4 boards accounted for 71.3% of the total losses, indicating that the main contention point is also in the top 4 boards. The round yielded 58 points, with a percentage of 73.4%, and plate 4 produced 79 points, with a percentage of 46%. Through the scoring data of the board order, it can be determined that the woman's connection between the man's serve is restricted, so more direct scores are formed, but this does not indicate that the woman's overall receiving effect is good because it is at a relative disadvantage in the 4 and 6 boards in this round.

The scoring rate of female receiver rounds was 48%. The results of multiple comparisons showed that female receiver rounds had significant differences from the four rounds with higher scoring rate, such as female receiver rounds and male receiver rounds, which belongs to the weakest round in different receiver rounds. The shots are women's 2, men's 4, women's 6, women's serve, men's 3, women's 5, and so on. The gain and loss points in the first 6 boards accounted for 82.8% of the total score in the round, with 56 points, 71.4%, boards 4 and 6, 101 and 38 points, respectively, and the score rate of 38.8% and 34.4%, respectively. The phenomenon of gain and loss of this round is very similar to the female receiving male round, especially the 4, 6 board loss phenomenon is more obvious, the phenomenon is produced because the other side of the man's third board attack quality and control ability is higher than that of women. Men are usually more active in mixed doubles, so when the shot of the men's third board plays the game, it poses a direct threat to the connection of the fourth and sixth boards. Through the data of this round, it is once again shown that the women's receiving wheel is obviously inferior in the 2 and 4 boards and after, and the fundamental reason for the weak women's receiving round is also found.

## 4. Construction of the Model of the Contribution of Male and Female Athletes to the Competition in Different Rounds

### 4.1. Concept Definition

Considering that a player has scoring behavior while losing points behavior in the game, the player's contribution is not measured only by “scoring rate” or “losing rate.” Both scoring behavior and loss behavior are considered. The score is regarded as the “positive contribution” to the game, the missing score is regarded as the “negative contribution” to the player, and the contribution to the game is compared through the size of the “absolute score.”

(2) $$\begin{array}{c} \text{Calculation of absolute score}:\text{absolute score}=\text{total score}-\text{total score.} \end{array}$$

The contribution of the male and female athletes to the competition in different rounds is analyzed by the mathematical method of multiple linear regression in two models.

### 4.2. Establishment of the First Regression Model

After observation and statistical analysis of the data, it was found that in different boards (first board, second board, third board, etc.). There are certain rules and differences between the gain and loss of male and female athletes. The relationship between absolute scores and total absolute scores between male and female athletes was analyzed using multiple linear regression.

#### 4.2.1. Model Establishment

Independent variables: absolute scores of the first, second, third, fourth, fifth, sixth (and after), and those of the first, second, third, fourth, fifth, sixth (and after), respectively, represented by *x*_*1*_*, x*_2_,…*,x*_12_; dependent variable: total absolute score for each game, indicated with *y*.  Table 4 shows the results of the model 1 regression coefficient calculation.

The regression analysis obtained the relationship between the independent variable and the dependent variable as follows:

(3) $$\begin{array}{c} Y=\sum_{i=1}^{12}\beta_{i}X_{i}. \end{array}$$

#### 4.2.2. Model Effectiveness Analysis

Analyzing the regression coefficient, we can see that the regression coefficient estimates are positive and negative, indicating that the absolute scores of different male and female athletes contribute differently to the total absolute scores. The coefficient of determination *R*^2^ = 0.3784 was calculated, indicating that 37.84% of the total amount of change in the dependent variable can be determined by the independent variable, indicating that the independent variable of this model could not explain the dependent variable very well. When *p*=0.9446, much larger than 0.05, this indicates that the regression model is very effective. The model needs to be improved before the regression analysis.

### 4.3. Construction of the Second Regression Model

Linear regression analysis of the total absolute score in 8 cases. In 8 cases, the absolute score of male and female athletes together, with *x*_1_, *x*_2_,…, *x*_8_ as dependent variable: Total absolute score is represented with *y*. The regression coefficients and confidence intervals calculated are shown in Table 5.

It can be seen from the table that the analytical regression coefficient estimates are positive and negative, indicating that the common absolute scores of male and female athletes contribute differently to the total absolute scores in different situations. Overall, the positive contribution is the big and the negative contribution. From the perspective of service, the regression coefficient was the largest, 1.7046, indicating that the joint score of men and women has the greatest impact on the results. In the corresponding female and male case, the regression coefficient was −0.3504, indicating that the joint score of men and women does not contribute much to the results and is negative. For male males, the regression coefficient was −0.3908, indicating that the combined score contributed contribute much to the results and is similar to that of female males. In female cases, the regression coefficient was 0.98227, indicating that the combined score contributed more to the results, but was less influential than in female men. It can be said that from the point of view of serving, male athletes serve more points, that is, more dominant.

As can be seen from Figure 5, from the perspective of receiving, the regression coefficient is 0.8969, which indicates that the joint score of men and women has a great influence on the results. In the corresponding female receiver, the regression coefficient is 0.6804, which indicates that the common score of men and women also makes a great contribution to the results, but no male receiver. For the male receiver, the regression coefficient is −0.5227, which indicates that the joint score between men and women does not contribute much to the results and is negative, while for the female receiver, the regression coefficient is 0.2402, which indicates that the joint score does not contribute much to the results, but it is a positive effect. It can be said that from the perspective of receiving, the score difference between male and female players is not very big, but female players may be more stable in receiving ball.

The model validity analysis calculated the determination coefficient *R*^2^ = 0.5922, which indicates that the proportion of the dependent variable is large; that is, the independent variable plays a large role in the dependent variable. With *p*=0.0641, close to 0.05, the model works well overall.

### 4.4. Study Conclusion

The above two models analyze the regression coefficients from different aspects, and we can see that the regression coefficient estimates are positive and negative, indicating that the common absolute scores of male and female athletes contribute differently to the total absolute scores in different cases. From the point of view of serving, male athletes serve more points, that is, more dominant. From the receiving point of view, the score difference between men and women is not very great, but female players may be more consistent. From the value of statistics *R*^2^ and *p*, the contribution of male and female scores to the game is more effective than model 1 and model 2 for different rounds. Therefore, model 2 is more efficient in the analysis of high-level table tennis competitions.

This study introduces the application of multiple regression analysis in table tennis mixed doubles. In subsequent studies, deep analysis and discussion of singles or doubles [20–24]. Besides, in practice, in commercial, construction, or other sports games, it can solve many practical problems.

## Figures and Tables

**Figure 1:** Eight rounds of mixed doubles competition.

**Figure 2:** Rate of different rounds in mixed doubles.

**Figure 3:** Contribution rate of service rounds.

**Figure 4:** Rate of gain and loss between men and women.

**Figure 5:** Linear regression analysis of common absolute versus total absolute scores between male and female athletes.

**Table 1:** Observation times of 20 table tennis mixed doubles matches.

The number of showings of a film	Score	The number of showings of a film	Score
2018 Austrian open final	3 : 2	2019 Korea open mixed doubles semifinals	3 : 1
2019 Swedish open mixed doubles final	3 : 2	2019 Qatar open mixed doubles final	3 : 0
The 2020 German open mixed doubles final	3 : 1	Mixed doubles semifinals at the 2019 Asian championships	3 : 2
Mixed doubles final at the 2017 Asian championships	3 : 1	Mixed doubles quarterfinals of the 55th world table tennis championships	4 : 3
Mixed doubles semifinals at the 2018 Asian games	4 : 0	2019 mixed doubles quarterfinals of the Qatar open	4 : 2
Mixed doubles semifinals at the 2018 Asian games	4 : 1	Mixed doubles final of the 54th world table tennis championships	4 : 1
Mixed doubles final at the 2018 Asian games	4 : 0	Mixed doubles final of the 55th world table tennis championships	4 : 3
Mixed doubles final at the 2019 Asian championships	3 : 1	2019 international table tennis federation finals mixed doubles final	4 : 1
The 2018 Austrian open mixed doubles quarterfinals	4 : 1	Mixed doubles semifinal of the 55th world table tennis championships	4 : 0
2019 Korea open mixed doubles final	4 : 1	2019 ITTF finals semifinal	3 : 0

**Table 2:** Statistics of service rounds.

Total serve score	Total loss of serve	Male score	Men lost points	Score rate for men	Male loss rate	Female score	Female hair lost points	Score rate for female hair	Female score loss rate
29	16	12	8	41.38%	50.00%	17	8	58.62%	50.00%
24	20	12	9	50.00%	45.00%	12	11	50.00%	55.00%
23	22	10	10	43.48%	45.45%	13	12	56.52%	54.55%
45	25	19	13	42.22%	52.00%	26	12	57.78%	48.00%
22	15	11	7	50.00%	46.67%	11	8	50.00%	53.33%
37	30	16	14	43.24%	46.67%	21	16	56.76%	53.33%
32	17	18	10	56.25%	58.82%	14	7	43.75%	41.18%
19	10	9	4	47.37%	40.00%	10	6	52.63%	60.00%
19	18	12	8	63.16%	44.44%	7	10	36.84%	55.56%
25	16	9	9	36.00%	56.25%	16	7	64.00%	43.75%
27	21	10	12	37.04%	57.14%	17	9	62.96%	42.86%
29	19	14	8	48.28%	42.11%	15	11	51.72%	57.89%
16	24	5	12	31.25%	50.00%	11	12	68.75%	50.00%
24	13	10	6	41.67%	46.15%	14	7	58.33%	53.85%
22	14	10	6	45.45%	42.86%	12	8	54.55%	57.14%
38	27	16	13	42.11%	48.15%	22	14	57.89%	51.85%
23	22	10	11	43.48%	50.00%	13	11	56.52%	50.00%
20	6	8	3	40.00%	50.00%	12	3	60.00%	50.00%
12	11	6	6	50.00%	54.55%	6	5	50.00%	45.45%
24	14	10	6	41.67%	42.86%	14	8	58.33%	57.14%
			Average	44.70%	48.46%		Average	55.30%	51.54%

**Table 3:** Statistical table of receiving gains and losses.

Total score on catch	Total points lost from receiving the ball	Male score	Men lost points	Male score rate	Male score loss rate	Female score	Women loss points	Female score rate	Female score rate
24	21	14	8	58.33%	38.10%	10	13	41.67%	61.90%
20	26	10	13	50.00%	50.00%	10	13	50.00%	50.00%
28	16	13	9	46.43%	56.25%	15	7	53.57%	43.75%
25	35	12	18	48.00%	51.43%	13	17	52.00%	48.57%
18	19	8	12	44.44%	63.16%	10	7	55.56%	36.84%
33	32	15	12	45.45%	37.50%	18	20	54.55%	62.50%
23	22	14	12	60.87%	54.55%	9	10	39.13%	45.45%
25	10	13	4	52.00%	40.00%	12	6	48.00%	60.00%
23	17	17	6	73.91%	35.29%	6	11	26.09%	64.71%
19	22	11	8	57.89%	36.36%	8	14	42.11%	63.64%
19	29	10	15	52.63%	51.72%	9	14	47.37%	48.28%
21	24	13	9	61.90%	37.50%	8	15	38.10%	62.50%
23	17	10	9	43.48%	52.94%	13	8	56.52%	47.06%
17	20	8	10	47.06%	50.00%	9	10	52.94%	50.00%
20	16	11	8	55.00%	50.00%	9	8	45.00%	50.00%
34	35	14	21	41.18%	60.00%	20	14	58.82%	40.00%
22	21	11	9	50.00%	42.86%	11	12	50.00%	57.14%
15	9	10	3	66.67%	33.33%	5	6	33.33%	66.67%
15	8	7	4	46.67%	50.00%	8	4	53.33%	50.00%
19	20	10	10	52.63%	50.00%	9	10	47.37%	50.00%
			Average	52.73%	47.05%		Average	47.27%	52.95%

**Table 4:** Results of the model 1 regression coefficient calculation.

Regression coefficient	Regression coefficient estimates	Confidence interval of the regression coefficient
*β *_0_	−3.3462	[−26.0158, 19.3234]
*β *_1_	1.3767	[−3.7309, 6.4844]
*β *_2_	0.7549	[−1.6929, 3.2027]
*β *_3_	0.7645	[−1.2041, 2.7331]
*β *_4_	0.7436	[−1.7025, 3.1897]
*β *_5_	−1.2333	[−5.4248, 2.9581]
*β *_6_	0.6579	[−1.8865, 3.2024]
*β *_7_	2.0006	[−2.7307, 6.7318]
*β *_8_	0.7568	[−1.6737, 3.1873]
*β *_9_	0.6576	[−1.9490, 3.2642]
*β*10	2.4270	[−1.5715, 6.4256]
*β*11	1.7717	[−4.0662, 7.6096]
*β*12	0.1402	[−4.0191, 4.2995]

*R * ^*2*^ = 0.3784, *F* = 0.3551, *p*=0.9446, *s*^2^ = 85.0852		

**Table 5:** Results of the regression coefficients calculated for the second model.

Regression coefficient estimates	Confidence interval
Of the regression coefficient	
−0.3908	[−1.6656, 0.8840]
1.7046	[0.3707, 3.0385]
−0.3504	[−1.7046, 1.0038]
0.9823	[−0.2252, 2.1897]
0.8969	[−1.7355, 3.5293]
−0.5226	[−3.1351, 2.0898]
0.2402	[−1.1250, 1.6054]
0.6805	[−0.7206, 2.0816]

## Data Availability

The data used to support the ﬁndings of this study are available from the corresponding author upon request.
